The article "Pan-Logical Probabilistic Algorithms Based on Convolutional Neural Networks" was retracted in 2023. Reasons: signs of a paper mill; suspected computer-generated content; unreliable results or conclusions; concerns about the data.

# Pan-Logical Probabilistic Algorithms Based on Convolutional Neural Networks

**DOI:** 10.1155/2022/8935906

**Published:** 2022-08-10

**Authors:** Fangrong Liu

**Affiliations:** School of Marxism Studies, Chongqing University of Education, Chongqing 400025, China

## Abstract

A brand-new kind of flexible logic system called universal logic aims to address a variety of uncertain problems. In this study, the role of convolutional neural networks in assessing probabilistic pan-logic algorithms is investigated. A generic logic probability algorithm analysis based on a convolutional neural network is suggested due to the unpredictable outputs of the probabilistic algorithm and the difficulty of its analysis. The stochastic gradient descent technique and the error backpropagation algorithm are used to investigate the broad logic probability algorithm (SGD). The experimental data presented in this research show that the BP algorithm of the convolutional neural network has an accuracy rate of 89 percent when analysing the experimental data. As there are more experimental iterations, the error will go down. The SGD method proves that raising the algorithm's learning rate reduces the loss value of the function. The loss value can be as low as 100%, and the algorithm analysis is closer to the real.

## 1. Introduction

There are more than a dozen well-known uncertainty inference models. However, because it generally specifies a variety of logical expressions and rules based on subjective experience, and also lacks feasibility and rationality analysis, its blindness and randomness are strong, so its application is not extensive. Therefore, the new system of pan-logic is introduced, which is a theory of uncertainty reasoning based on the thinking and experience of human past experience and on the basis of thinking with real experience.

In the scientific community, the logic system will have important academic significance and practical value not only in probabilistic logic but also in various probability-based uncertainty reasoning methods. The basic function of probabilistic algorithms is that solving the same instance of a problem twice using the same probabilistic algorithm can produce completely different results. It can take a long time to get a wrong answer. It also can take a very short time to calculate the optimal solution. A clear understanding of the pan-logical probabilistic algorithms can help one increase the correct rate of random selection when the correct result is not available or difficult to obtain.

A convolutional neural network is suggested in this paper to analyse the pan-logic probability algorithm. Experiments comparing the accuracy and data convergence of the original analysis method and the addition algorithm analysis method led to the conclusion that the addition algorithm can increase analysis accuracy and quicken convergence. In order to achieve the experimental results, the BP algorithm in this paper innovates by continuously adjusting the BP network, calculating the error, and reversing the weight according to the error. The minimum loss function value is then calculated by the SGD algorithm, which lowers the experimental error by first calculating the gradient of the loss function.

The article "Pan-Logical Probabilistic Algorithms Based on Convolutional Neural Networks" was retracted in 2023. Reasons: signs of a paper mill; suspected computer-generated content; unreliable results or conclusions; concerns about the data.

## 2. Related Work

A potent strategy for resolving the continuous variables of various operators with unclear reasoning has emerged with pan-logic. Related works on the pan-logic probability algorithm include the following: Frieze and Tkocz [1] investigated the probabilistic analysis of the least-weighted combinatorial object algorithm. In response to the difficulties in medical image analysis, Yang et al. [2] suggested a novel multimodal medical image fusion method based on SPD and pan-logic methodologies. Lin developed a new clustering approach by applying correlation coefficient formulas to analyse the links between two sets of probabilistic language phrases. Current tracking techniques are unreliable because target templates are utilised to represent target candidates. Wei et al. consequently obtained the foundation from the probability matrix decomposition in order to collect the goal structural information and local information. In order to address the problem of information overload in the use of e-government systems and suit users' specific demands, Xu et al. suggested a personalised e-government recommendation algorithm that combines probabilistic semantic clustering analysis and collaborative filtering [3]. The linked study currently concentrates primarily on the application of probabilistic algorithms, and the related analysis work is currently comparatively immature. The convolutional neural network is introduced to analyse and summarise the pan-logic probability method.

Convolutional neural networks have been the subject of related study by the following scientists: To solve the problem that most current approaches cannot extract great centerline networks that look smooth, full, and single-pixel wide, Cheng et al. developed cascaded end-to-end convolutional neural networks for road detection and centerline detection [4]. Lee et al. presented the FDC-CNN network model [5] to extract fault features for the receptive field optimised for multivariate sensor signals sliding along the time axis. In order to address the issue of the time-consuming, arduous, and subjective inspection of nuclear power plants, several scholars have proposed a data fusion strategy using NB-CNN to increase the overall performance and resilience of the system [6]. Because the transition from low spatial resolution MS images to high spatial resolution MS images is difficult and extremely nonlinear, Yuan et al. suggested a multi-scale and multi-depth CNN for panchromatic sharpening of remote sensing images [7]. For the identification of multimodal and multidimensional facial expressions, Li et al. investigated a unique DF-CNN [8]. However, more research is needed in this field because convolutional neural networks are only better at identifying characteristics, not interpreting them.

The article "Pan-Logical Probabilistic Algorithms Based on Convolutional Neural Networks" was retracted in 2023. Reasons: signs of a paper mill; suspected computer-generated content; unreliable results or conclusions; concerns about the data.

## 3. Deconstruction Method of Pan-Logical Probabilistic Algorithm Based on Convolutional Neural Network

### 3.1. Pan-Logical Probabilistic Algorithms

In life and teaching experiments, problems such as definite integrals or nonlinear equations and problems with uncertain answers are often encountered in life. At this time, probability algorithms can be applied. It allows people to randomly select one of the possible answers. Compared with insisting on calculating the correct answer, this randomness with a tentative optimal solution can reduce the time and space complexity of the algorithm. The randomness in this algorithm greatly improves the flexibility of algorithm design and the possibility of people solving problems. But because of the wide range of random selection, the accuracy rate is not very high [9].

Pan-logic is mainly to study the common laws between flexible logic and mathematical logic. In pan-logic, correlation is introduced to describe that all things in the world are related to each other. One of the biggest features of probabilistic algorithms is that using the same method to solve the same problem may end up with completely different results. Similar to the Las Vegas probabilistic algorithm, using its similar random properties can help speed up analytical problem solving. For some unsolved problems for which a suitable algorithm has not yet been found, a probabilistic algorithm can also be used to roughly find a solution.

Usually, probabilistic logic systems provide these three independent operators, but the implicit operators are not clearly defined and are often treated as conditional probabilities. The analysis of these random theorem operators based on general logic principles reveals the following main problems:

1. The generalized correlation coefficient affects the probability logic operator and makes flexible changes according to the change of the correlation coefficient. However, traditional random operators do not consider the influence of general correlation, and the presented logical relationship is rigid.
2. The definition of conditional probability takes into account independence but makes no connection between independence and conditional probability.
3. In uncertainty reasoning, conditional probability is often regarded as a constant, which is obviously unreasonable, and the conditional probability should not be a constant.
4. The expression of conditional probability does not correspond to the logical expression, and conditional reasoning cannot be done because the same definition of conditional probability cannot be given in probability space.

The article "Pan-Logical Probabilistic Algorithms Based on Convolutional Neural Networks" was retracted in 2023. Reasons: signs of a paper mill; suspected computer-generated content; unreliable results or conclusions; concerns about the data.

The above problems seriously affect the application of the general logic probability algorithm. Therefore, a convolutional neural network is introduced to analyse the probability algorithm and to establish a related model, so that the logical relationship representing flexibility and rigidity can be realized.

### 3.2. Application of Convolutional Neural Network in Probabilistic Algorithm in Pan-Logic

Convolutional neural networks can reduce the number of weights that need to be learned and the complexity of network computation by adjusting the weight distribution. Downsampling ensures the invariance of the network in terms of the local transformations returned and improves the generalization ability of the network. Among them, the analysis and research of the probabilistic algorithm of pan-logic is mainly applied to the BP algorithm and the SGD algorithm in the convolutional neural network.

#### 3.2.1. A Technique for Using the BP Algorithm to Analyse the General Logic Probability Algorithm

The BP network is one of the most widely used neural network models in machine learning algorithm models [10–12]. It has three layers: an input layer, a hidden layer and an output layer. It is a forward multi-layer network. An error propagation algorithm governs it. Despite layers one through three being virtually totally connected, there is no connection between cells within the same layer; however, there is no connectivity between cells within the same layer. When training samples carry the network, neural activations diffuse from the input layer to the output layer. After receiving network input responses from the neurons in the intermediate and output layers, each connection weight of each layer of the output layer changes in line with the direction. Before returning to the input layer, the error backpropagation method, also referred to as the BP algorithm, passes through each intermediate layer in an effort to reduce the error between the desired output and the output.

The BP network's basic working principle is to map the input space to the output space by converting the input vector into the output vector through the hidden layer. Utilizing weights discovered by contrasting the network's actual output with what would be predicted based on the behaviour of the current weights, forward mapping is carried out. The network uses the actual error to modify the weights in order to lower the overall error. Because assembling a team to train the model necessitates the anticipated output correlating to the input, the BP network must direct learning.

The article "Pan-Logical Probabilistic Algorithms Based on Convolutional Neural Networks" was retracted in 2023. Reasons: signs of a paper mill; suspected computer-generated content; unreliable results or conclusions; concerns about the data.

The BP network's structure is symmetrical, and each output processing unit has essentially the same transmission function, as forming a training mode team requires the expected output to match the input.  Figure 1 depicts the BP algorithm's network structure diagram:

Figure 1 depicts the relationships between the input layer, hidden layer and output layer in the BP algorithm. Every neuron in the BP algorithm may be derived, regardless of when and where it appears in the transfer function. Each layer of neurons in the BP network, including the log-sigmoid function and the tan-sigmoid function, adopts the sigmoid transfer function. The input value of (−*∞*, +*∞*) is mapped to (0,1) and (−1, +1), respectively, and the mapping effect of the two transfer functions is shown in Figure 2:

Backpropagation is used to determine the error function: *n* learning samples are input, denoted by *x*^1^, *x*^2^,…*x*^*n*^ respectively. The corresponding output is represented by *y*_*i*_^*n*^  (*i*=1,2,…*m*), and the squared error function is used to obtain the error *E*_*n*_ of the *n*th sample. Its expression is defined as formula (1):

(1) $$\begin{array}{c} E_{n}=\frac{1}{2}\sum_{i=1}^{m}{\left(t_{i}^{n}-y_{i}^{n}\right)}^{2}. \end{array}$$

In formula (1), *t*_*i*_^*n*^ represents the desired output.

For *n* samples, the global error expression is defined as formula (2):

(2) $$\begin{array}{c} E=\frac{1}{2}\sum_{n=1}^{n}\sum_{i=1}^{m}{\left(t_{i}^{n}-y_{i}^{n}\right)}^{2}\\ =\sum_{n=1}^{n}E_{n}. \end{array}$$

There are changes in the weights of the backpropagation output layer: The cumulative error BP algorithm is used to adjust *w*_*ik*_ to make the global error value smaller. Its expression is defined as formula (3):

(3) $$\begin{array}{c} \Delta w_{ik}=-\vartheta \frac{\partial E}{\partial w_{ik}}\\ =-\vartheta \frac{\partial }{\partial w_{ik}}\left(\sum_{n=1}^{n}E_{n}\right)\\ =\sum_{n=1}^{n}\left(-\vartheta \frac{\partial E_{n}}{\partial w_{ik}}\right). \end{array}$$

In formula (3), 0 < *ϑ* < 1, which represents the learning rate. *E*_*n*_ represents the error of the *n*th sample and *∂E*_*n*_ represents the derivative of the error.

The error signal is defined as formula (4):

(4) $$\begin{array}{c} \delta_{yi}=-\frac{\partial E_{n}}{\partial S_{i}}\\ =-\frac{\partial E_{n}}{\partial y_{i}}\cdot \frac{\partial y_{i}}{\partial S_{i}}. \end{array}$$

Among them, there are formulas (5) and (6):

(5) $$\begin{array}{c} \frac{\partial E_{n}}{\partial y_{i}}=\frac{\partial }{\partial y_{i}}\left[\frac{1}{2}\sum_{i=1}^{m}{\left(t_{i}^{n}-y_{i}^{n}\right)}^{2}\right] \end{array}$$

(6) $$\begin{array}{c} \frac{\partial y_{i}}{\partial S_{i}}=f_{2}^{\prime }\left(S_{i}\right). \end{array}$$

Finally, the weight formula of each neuron in the output layer is adjusted, which is adjusted as formula (7):

(7) $$\begin{array}{c} \Delta w_{ik}=\sum_{n=1}^{n}\sum_{i=1}^{m}\vartheta \left(t_{i}^{n}-y_{i}^{n}\right)f_{2}^{\prime }\left(S_{i}\right)\cdot z_{k}. \end{array}$$

Backpropagation of changes in hidden layer weights is defined as formula (8):

(8) $$\begin{array}{c} \Delta v_{ki}=-\vartheta \frac{\partial E}{\partial v_{ki}}\\ =-\vartheta \frac{\partial }{\partial v_{ki}}\left(\sum_{n=1}^{n}E_{n}\right)\\ =\sum_{n=1}^{n}\left(-\vartheta \frac{\partial E_{n}}{\partial v_{ki}}\right). \end{array}$$

The error signal is defined as formula (9):

(9) $$\begin{array}{c} \delta_{zk}=-\frac{\partial E_{n}}{\partial S_{k}}\\ =-\frac{\partial E_{n}}{\partial z_{k}}\cdot \frac{\partial z_{k}}{\partial S_{k}}. \end{array}$$

Among them, formula (10) can be obtained:

(10) $$\begin{array}{c} \frac{\partial E_{n}}{\partial z_{k}}=\frac{\partial }{\partial z_{k}}\left[\frac{1}{2}\sum_{i=1}^{m}{\left(t_{i}^{n}-y_{i}^{n}\right)}^{2}\right]\\ =-\sum_{i=1}^{m}\left(t_{i}^{n}-y_{i}^{n}\right)\frac{\partial y_{i}}{\partial z_{k}}. \end{array}$$

From the chain theorem, formula (11) can be obtained:

(11) $$\begin{array}{c} \frac{\partial y_{i}}{\partial z_{k}}=\frac{\partial y_{i}}{\partial S_{i}}.\frac{\partial S_{i}}{\partial z_{k}}\\ =f_{2}^{\prime }\left(S_{i}\right)w_{ik}. \end{array}$$

Finally, the weight adjustment formula of each hidden neuron is obtained as formula (12):

(12) $$\begin{array}{c} \Delta v_{ki}=\sum_{n=1}^{n}\sum_{i=1}^{m}\vartheta \left(t_{i}^{n}-y_{i}^{n}\right)f_{2}^{\prime }\left(S_{i}\right)w_{ik}f_{1}^{\prime }\left(S_{k}\right)\cdot x_{i}. \end{array}$$

The training of the BP algorithm is a complex process. It is necessary to continuously adjust the BP network according to the training samples, continuously calculate the error and reversely adjust the weight according to the error. The method of adjusting the weights in this paper incorporates the law of stochastic gradient descent to introduce information such as the input value of the direct input. The chain rate is used to obtain a faster and more accurate weight update method, which enables the BP neural network to obtain better training results. Among them, the gradient descent method is an important part of the delta law [13]. It uses the descent method to search for potential weight vectors to obtain the best fit training effect and provide the best learning effect.

The article "Pan-Logical Probabilistic Algorithms Based on Convolutional Neural Networks" was retracted in 2023. Reasons: signs of a paper mill; suspected computer-generated content; unreliable results or conclusions; concerns about the data.

#### 3.2.2. Application Method of SGD Algorithm in the Analysis of the Probability Algorithm of General Logic

The SGD algorithm's central premise is to first determine the loss function's slope. By continuously modifying the weights, the optimal solution problem is solved, and the loss of the function is minimised in accordance with the trend of the slope, resulting in the minimum loss value of the function. Because only one sample is randomly chosen and updated each time rather than all samples, SGD drastically reduces the computational complexity and saves a lot of time [14]. SGD is favoured by many researchers because of its easy convergence and fast training speed, and it has become their most commonly used optimization algorithm. Its related formula is defined as formula (13):

(13) $$\begin{array}{c} g\left(\omega \right)=\sum_{i=0}^{n}\omega_{i}x_{i}. \end{array}$$

In formula (13), *ω* represents the parameter weight and *g*(*ω*) represents the objective function.

(14) $$\begin{array}{c} h\left(\omega \right)=\frac{1}{2m}\sum_{j=1}^{m}{\left(y_{j}-g_{\omega }\left(x^{j}\right)\right)}^{2}. \end{array}$$

In formula (14), *y*_*j*_ represents the sample value of the *j*th sample and *h*(*ω*) represents the loss function. *m* represents the total number of iterations of the formula for calculation.

(15) $$\begin{array}{c} \omega ≔\omega -\alpha \nabla_{\omega }h\left(\omega \right). \end{array}$$

In formula (15), *ω* represents the parameter weight; *α* represents the gradient descent step size, also known as the learning rate; ∇_*ω*_ represents the gradient. The learning rate is very important to the computation of the gradient descent algorithm. Setting it too low can result in more iterations to find the optimal solution, and even slow down the network convergence. Worse results are situations that also lead to stagnation of the local optimum. However, if the value of *α* is set too high, although it will speed up the training speed of CNN [15], and it also increases the possibility of skipping the optimal solution in the calculation, so that the optimal solution cannot be calculated in the end. It can be seen that the value of *α* is the key factor determining the computational efficiency of the algorithm, and the value should not be too large or too small when setting this value.

The stochastic gradient algorithm is an iterative algorithm that optimizes neural networks, and its purpose is to calculate partial gradients of random subsets of data, rather than the entire actual gradient. The expression for updating the weights with a series of small samples is defined as formulas (16) and (17):

(16) $$\begin{array}{c} w_{x+1}=w_{x}+\Delta w_{x}, \end{array}$$

(17) $$\begin{array}{c} \Delta w_{x}=-\eta \nabla_{w}E\left(w_{x}\right). \end{array}$$

Among them, *η* represents the algorithm learning rate; *E*(*w*_*x*_) represents the loss function of the *x*th iteration weight *w*_*x*_; ∇_*w*_*E*(*w*_*x*_) represents the first-order gradient of the loss function when the weight *w* is at *x*. Δ*w* stands for the gradient operator, which is the part where the weights are updated at each iteration [16]. However, the stochastic gradient algorithm also has obvious shortcomings. It uses the same learning rate every time the weights are updated in each iteration. Therefore, when the analysis object is sparse data or sparse features, the result will be less than ideal. In addition, there are gradient noise and variance. The final optimization result of the stochastic gradient is given using the proximal stochastic gradient algorithm. Its optimised partial expression is defined as formula (18):

(18) $$\begin{array}{c} w_{x+1}={\text{prox}}_{\eta_{t\theta }}w_{x}-\eta_{x}\nabla \varphi_{i_{x}}\left(w_{x}\right). \end{array}$$

In formula (18), prox represents the near-end operator of the near-end stochastic gradient descent algorithm, from which *i*_*x*_ samples are randomly selected per iteration. The algorithm also has the disadvantage of instability. Based on this, the concept of momentum is introduced. When the weight parameters are updated, the previous update methods will remain unchanged to a certain extent, and the final method will be adjusted according to the current data [17]. Its algorithm expression is defined as formulas (19) and (20):

(19) $$\begin{array}{c} \Delta w_{x}=\rho \Delta w_{x-1}-\eta g_{x}, \end{array}$$

(20) $$\begin{array}{c} w_{x}=w_{x-1}+\Delta w_{x}. \end{array}$$

In formulas (19) and (20), *ρ* is the momentum factor, which represents the number of degrees to retain the original update direction. The momentum factor extends the update range and recovers from a local optimum. If the direction of the slope is changed, the momentum factor is less updated. In general, the impulse element can accelerate the stochastic gradient algorithm in the appropriate direction, which can suppress oscillation, and accelerate convergence. The Adadelta algorithm is a one-dimensional learning gradient decreasing algorithm, which uses a similar momentum coefficient averaging algorithm. The algorithm update expression is defined as formulas (21)–(23):

(21) $$\begin{array}{c} E{\left[g^{2}\right]}_{x}=\rho E{\left[g^{2}\right]}_{x-1}+\left(1-\rho \right)g_{x}^{2}, \end{array}$$

(22) $$\begin{array}{c} \Delta w_{x}=-\frac{\eta }{\sqrt{E{\left[g^{2}\right]}_{x}+\varepsilon }}, \end{array}$$

(23) $$\begin{array}{c} w_{x}=w_{x-1}+\Delta w_{x}. \end{array}$$

In formulas (21)–(23), *E* is the expectation; *ρ* is the exponential decay rate; *ε* is to prevent the denominator from being equal to 0.

The article "Pan-Logical Probabilistic Algorithms Based on Convolutional Neural Networks" was retracted in 2023. Reasons: signs of a paper mill; suspected computer-generated content; unreliable results or conclusions; concerns about the data.

## 4. Experimental Results of the Pan-Logic Probability Algorithm Based on Convolutional Neural Network

### 4.1. Experimental Results of BP Algorithm

The purpose of the analysis of the pan-logic probability algorithm based on the BP algorithm is that the relevant data of the algorithm analysis model is used as the training sample of the BP algorithm, and the BP neural network is used to train the data, so as to improve the probability algorithm and obtain the experimental results with higher accuracy. In the process of algorithm analysis and research, in addition to selecting experimental learning samples, verification samples should also be selected according to the samples. The two sample data are shown in Tables 1 and 2:

Tables 1 and 2 record the data of the experimental items, the actual number of wrong modules and the actual number of correct modules. In the experimental process of the probability algorithm research based on the BP algorithm, the input parameters of the BP algorithm are set according to the number of parameters of the experimental data itself. The parameters Ac, Pc and *R* of the evaluation prediction results are obtained through experiments, and the results are shown in Figure 3:

The experimental results demonstrate that when the BP algorithm is used for analysis and learning, the PC2 sample data set has the best prediction effect, with an accuracy rate of up to 89 percent. The accuracy of other sample data sets' predictions is at least 70%. This demonstrates that an algorithm analysis based on BP can forecast analysis accuracy based on sample data information and achieve a specific application-feasible prediction effect [18]. In fact, there is a strong correlation between the quantity of sample data and the quality of the prediction effect. The learning effect will be better the more sample data there are.  Figure 4 displays its experimental comparison chart.

During the experiment, a specific task of normalizing the training data is to summarise the statistical distribution of the integrated samples. For the alienation problem, the input samples are either 0 or 1, so the learning of the XOR problem does not require data normalization [19]. The training error curve of the standard BP algorithm is shown in Figure 5:

Figure 5(a) shows the grid training error curve of the standard BP algorithm, and it reaches the error accuracy after 218 cycles, while the adaptive learning rate BP algorithm in Figure 5(b) achieves the error accuracy after only 25 cycles. The comparison demonstrates that the adaptive learning rate algorithm takes far less training sessions than the traditional approach to obtain the same accuracy. This is primarily due to the adaptive learning rate algorithm's addition of a learning rate adaption factor. As a result, the network's weights and thresholds are also modified in real time, enabling it to swiftly approach the desired goal value. Convergence speed and accuracy are significantly influenced by the learning rate. The system may overcompensate and oscillate or diverge if the learning rate is too high, which would make the system unstable. The training period will be lengthy, and convergence will occur slowly, if the learning rate is too low. The aforementioned simulation results demonstrate that the learning rate adaptable coefficient-added algorithm has a superior convergence impact than the approach with a fixed learning rate.

The article "Pan-Logical Probabilistic Algorithms Based on Convolutional Neural Networks" was retracted in 2023. Reasons: signs of a paper mill; suspected computer-generated content; unreliable results or conclusions; concerns about the data.

### 4.2. Experimental Results of SGD Algorithm

Nowadays, all common CNN architectures add pulses to the SGD implementation, the purpose of which is to prevent the CNN from continuing to iterate at the point where the loss is minimal and ensure that it does not stall [20]. In this paper, in order not to drastically reduce the learning speed of the algorithm, a new learning speed rule is specially defined. According to the newly set learning rate rule, the learning rate will be updated from time to time with each calculation iteration, so the learning rate will also be updated accordingly from time to time. The loss value of the function gradually decreases as the number of iterations increases, and the learning rate also decreases accordingly. The trend is shown in Figure 6:

Figure 6 illustrates how the learning rate gradually declines as the number of repetitions rises. The greatest and minimum learning rates are around 0.17 and 0.01 respectively. There are several factors to consider when determining whether an algorithm is effective and performs effectively. The accuracy of the training set, the accuracy of the cross-test set and the convergence of the optimization method are just a few of the numerous factors that can be used to assess an algorithm's benefits and drawbacks. These three algorithm assessment standards are employed in this research to assess and examine the experimental algorithm. Figures 7 and 8 display the convergence outcomes after 200 iterations of the experimental process on the MNIST and CIFAR-10 datasets, respectively.

The article "Pan-Logical Probabilistic Algorithms Based on Convolutional Neural Networks" was retracted in 2023. Reasons: signs of a paper mill; suspected computer-generated content; unreliable results or conclusions; concerns about the data.

The three curves in the figure represent the change curves of the loss value of the training function and the loss value of the verification state under the running state of Relu, Leaky Relu and SGD activation functions respectively. The loss value of the training function is represented by train loss. The loss value of the validation function is represented by val-loss, and Epochs represent the total number of iterations in the calculation process [21]. It can be seen from Figure 8 that the more the iterations are, the smaller the loss value will be. The loss value of using the Relu activation function is not much different from the loss value of using the Leaky Relu activation function. There are overlapping parts, but the loss value is too large and the Leaky Relu activation function is used. The network loss value using the SGD algorithm is the smallest, which tends to be stable, and the network converges faster. It goes without saying that the network convergence of the SGD algorithm is a nonadaptive algorithm.

In addition, the number of algorithm iterations is related to the degree of heterogeneity. When the degree of heterogeneity increases, the number of iterations required will also increase.  Figure 9 displays the outcomes of the experiment:

The results demonstrate that when the degree of inconsistency grows from 1 to 2, the number of iterations varies as the algorithm approaches the predetermined error rate, hence lowering the number of iterations required to attain convergence. Because of this, each cycle can yield updates that are more effectively updated, bringing the global parameters even closer to the ideal outcome. The DASGD algorithm's iteration number increases less over the training phase, and the method's performance is also improved. The larger the number of iterations, the less effective the algorithm is to update. It demonstrates how the DASGD algorithm can detect cluster delays and reduce the impact of excessive delays on global parameters to reduce the number of erroneous updates.

## 5. Conclusions

In the context of pan-logic, probabilistic algorithms address the issue of uncertain reasoning brought on by randomness from the viewpoint of probability and address pan-shortcomings logics in the study of probability algorithms. The development of science and technology benefits greatly from the use of probabilistic algorithms, which are probability-based algorithms based on probability theory. By investigating various probabilistic algorithms and incorporating them into the framework of general logic, or by investigating both probabilistic algorithms and pan-logic and making full use of both, both have contributed to the development and refinement of both theories, making them more useful in uncertain reasoning. In order to further the study and analysis of the general logic probability algorithm, convolutional neural networks will be used in this paper. The results of the experiment indicate that the convolutional neural network's BP algorithm has an accuracy rate of 89 percent when analysing the results. The experiment's error decreases with the number of iterations. The SGD algorithm demonstrates how increasing the algorithm's learning rate can lower the function's loss value. The algorithm analysis is more accurate and the loss value can be as low as. This makes it possible for people to fully comprehend probability algorithms and apply them to more technologies, thereby advancing science, technology and society [22].

The article "Pan-Logical Probabilistic Algorithms Based on Convolutional Neural Networks" was retracted in 2023. Reasons: signs of a paper mill; suspected computer-generated content; unreliable results or conclusions; concerns about the data.

## Figures and Tables

**Figure 1:** Network structure diagram of BP algorithm.

**Figure 2:** Transfer function mapping renderings. (a) Log-sigmoid function. (b) Tan-sigmoid function.

**Figure 3:** Prediction and analysis results of BP algorithm on the experimental results of probabilistic algorithm.

**Figure 4:** Relationship between sample size and R value.

**Figure 5:** Grid training error line.

**Figure 6:** Learning rate change curve.

**Figure 7:** Convergence curves of different networks in MNIST.

**Figure 8:** Convergence curves of different networks in CIFAR-10.

**Figure 9:** The number of iterations required for the algorithm to reach the specified error rate.

**Table 1:** Learning sample information data table.

Name	Actual number of error modules	Actual correct number of modules
CM1	40	300
MC2	45	86
KC3	35	165
PC1	60	704
PC2	18	1636
PC3	140	1000

**Table 2:** Validation sample information data sheet.

Name	Actual number of error modules	Actual correct number of modules
CM1	40	283
MC2	45	85
KC3	35	159
PC1	60	681
PC2	18	730
PC3	136	946

## Data Availability

The data used to support the findings of this study are available from the author upon request.
